The article "Evaluation of Mindfulness Training Combined with Aerobic Exercise on Neurological Function and Quality of Life in Patients with Peripheral Neuropathy Type 2 Diabetes Mellitus" was published in 2022. Journal: Contrast Media Mol Imaging.

# Evaluation of Mindfulness Training Combined with Aerobic Exercise on Neurological Function and Quality of Life in Patients with Peripheral Neuropathy Type 2 Diabetes Mellitus

**DOI:** 10.1155/2022/7665483

**Published:** 2022-08-05

**Authors:** Ximei Weng, Shunqi Liao, Fang Wang, Han Wang, Ling Yang

**Affiliations:** ^1^Chengdu University of Traditional Chinese Medicine, Chengdu, Sichuan 610075, China; ^2^Hospital of Chengdu University of Traditional Chinese Medicine, Chengdu, Sichuan 610075, China

## Abstract

**Objective:**

To investigate the effect of mindfulness training on neurological function and quality of life in patients with type 2 diabetic peripheral neuropathy.

**Methods:**

This study selected 120 patients with type 2 diabetic peripheral neuropathy and randomly divided them into three independent subgroups according to different training methods: mindfulness meditation group (MM), aerobic exercise group (AE), and mindfulness combined with aerobic exercise group. (MMAE). The three groups were analyzed for SNCV and MNCV velocities, MAAS and TCSS scores, neurological symptom scores, neurological sign scores, and quality of life.

**Results:**

Before treatment, SNCV and MNCV were not significantly significant (*P* > 0.05), but after treatment, SNCV and MNCV were significantly higher, and the MMAE group changed more significantly (*P* < 0.05); before treatment, MAAS and TCSS scores were not significant (*P* > 0.05), but after treatment, MAAS scores were significantly higher, TCSS scores were significantly lower, and more significantly in MMAE; the difference was significant (*P* < 0.05); before treatment, there was no statistical significance of the neurological signs score (*P* > 0.05); after treatment, the neurological symptoms score and neurological signs score were significantly reduced, and the changes in the MMAE group were statistically significant (*P* < 0.05); there was no significant difference in the quality of life score before treatment (*P* > 0.05), and the quality of life score in the MMAE group was significantly increased (*P* < 0.05).

**Conclusion:**

Mindfulness training combined with aerobic exercise has an ideal therapeutic effect on patients with type 2 diabetic peripheral neuropathy, and has a very important role in improving the neurological function and quality of life of the patients. It is a safe and effective treatment method. Therefore, mindfulness training combined with aerobic exercise is worthy of promotion and application.

## 1. Introduction

Diabetic peripheral neuropathy (DPN) refers to some of the symptoms or signs associated with peripheral neuropathy in people with diabetes in the absence of other causes. This is a relatively common diabetes complication. According to statistics, its incidence rate is as high as 90%; early treatment and intervention are very important. In the existing treatment methods, Chinese and western medicines have obvious side effects, slow onset of effects, long courses of treatment, complicated operations, inconvenient decoction, and increasingly prominent gastrointestinal irritation, and some patients are difficult to adhere to for a long time. Acupuncture treatment is more effective. However, some patients' fear of needles limits the application of acupuncture in the long-term treatment of DPN to a certain extent. Aerobic exercise combined with mindfulness training is safe and effective.

The article "Evaluation of Mindfulness Training Combined with Aerobic Exercise on Neurological Function and Quality of Life in Patients with Peripheral Neuropathy Type 2 Diabetes Mellitus" was published in 2022. Journal: Contrast Media Mol Imaging.

This study included 120 patients with type 2 diabetic peripheral neuropathy who underwent mindfulness meditation and Tai Chi training. The therapeutic effects of the two treatment methods are now analyzed, and the report is as follows.

## 2. Materials and Methods

### 2.1. General Information

This study selected 120 patients with type 2 diabetic peripheral neuropathy and randomly divided them into three independent subgroups according to different training methods: mindfulness meditation group (MM), aerobic exercise group (AE), and mindfulness combined with aerobic exercise group (MMAE). There were 120 patients, including 75 males and 45 females, aged 20–73 years, with an average age of 42.69 ± 3.8 years. The patients in this study were aware of the relevant content of the study and were approved by the hospital's ethics committee.

#### 2.1.1. Inclusion Criteria

1. Aged 45–75 years old, male or female
2. In accordance with the diagnostic criteria for DPN in the 2017 edition of the Chinese Guidelines for the Prevention and Treatment of Type 2 Diabetes
3. Muscle strength ≥ III grade and can complete moderate-intensity load exercise
4. Have not participated in systematic aerobic exercise exercises and mindfulness training before joining the group
5. No other adjuvant or comprehensive therapeutic approaches were used to intervene in DPN during the study
6. Clear consciousness, normal hearing, able to communicate with people normally, and able to understand and follow demonstration actions
7. Patients or their legal guardians sign the informed consents

#### 2.1.2. Exclusion Criteria

1. Patients with severe infection, severe heart, kidney, and other organ dysfunction, autoimmune diseases, and other neuroendocrine diseases
2. Hematological patients with bleeding tendency
3. Patients with severe osteoporosis or other exercise contraindications
4. Patients with diabetic foot ulcers or amputations
5. Women during pregnancy or breast feeding
6. Patients refuse to cooperate or mentally unable to cooperate, participants' withdrawal, dropout, and termination criteria.

The article "Evaluation of Mindfulness Training Combined with Aerobic Exercise on Neurological Function and Quality of Life in Patients with Peripheral Neuropathy Type 2 Diabetes Mellitus" was published in 2022. Journal: Contrast Media Mol Imaging.

### 2.2. Methods

#### 2.2.1. The Control Group

Patients in the control group do not receive any form of regular exercise but regular health education. Health education has been conducted every month centrally by the members of the study and consisted mainly of instruction on diabetic diet, exercise, medications, glucose monitoring, foot care, and prevention and treatment of foot complications After the first activity, a health education training booklet will be distributed to the participants.

#### 2.2.2. Aerobic Exercise Group (AE)

Patients in the aerobic exercise group (AE) will receive routine nursing, and aerobic training and aerobic exercise will be performed every Monday, Wednesday, and Friday. Aerobic exercise using the rowing machine or cycling, moderate-intensity training exercise (65–85% of the maximum heart rate) to ensure that the patient's heart rate is stable during exercise (120–150 times/min), and each group of training exercise time is 30 minutes.

#### 2.2.3. Mindfulness Meditation Combined with Aerobic Exercise group (MMAE)

Mindfulness meditation combined with aerobic exercise will be added on the basis of routine health education, and group intervention will be used in combination with mindfulness training, WeChat or telephone follow-up, consultation, and on-site guidance. Use mindfulness training based on “meta-awareness” combined with an attitude of control and acceptance of attention and reactive flexibility, dynamic self, and reflection on values. The national second-level psychological counselor and members of the research group who have been trained in mindfulness training technology are responsible for group intervention in the community. Group mindfulness training combined with aerobic exercise practice will be given 3 times a week, 1 to 1.5 hours each time. On nongroup training days, patients will be practicing mindfulness at home for 45 minutes every day, their experiences will be recorded and they will communicate with each other in WeChat groups or during group training. Team members will give timely feedback in order to integrate mindfulness into the subjects' daily life. The specific arrangement of the training is shown in Table 1.

### 2.3. Observation Indicators

#### 2.3.1. Nerve Conduction Velocity Testing (NCV)

*(1) Mindful Attention Awareness Scale (MAAS)*. The Mindful Attention Awareness Scale (MAAS) is a one-dimensional scale, involving a total of 15 items in the aspects of cognition, emotion, and physiology of individuals in daily life. In the test, the research subjects were asked to choose the most suitable description level in each item according to their actual situation in the last week. Each item is assigned a score of 1–6, with a scale ranging from “almost always” to “almost never”, with higher scores indicating higher levels of awareness and attention to the present.

*(2) Toronto Clinical Score (TCSS)*. Toronto Clinical Scoring (TCSS) is a scoring system developed by diabetes and neuropathy experts at the University of Toronto in 2001. TCSS scores include symptom scores, reflex scores, and sensory test scores. Among them, symptom score: yes = 1, no = 0; reflex score: no = 2, weakened = 1, normal = 0; sensory test score: abnormal = 1, normal = 0. The total TCSS score is 19 points, and the symptom evaluation is attributed to the total score. 6 points out of the total score, the reflex evaluation of both lower extremities is classified into 8 points out of the total score, and the sensory test evaluation of the thumb is classified into 5 points out of the total score. The lowest score is 0 and the highest score is 19, with higher scores indicating more severe symptoms.

*(3) Michigan Neuropathy Screening Instrument (MNSI)*. The Michigan Neuropathy Screening Instrument (MNSI) was proposed in 1994. The MNSI score includes two parts, A and B. Among them, part A 1–3, 5–6, 8–9, 11–12, and 14–15 answer yes 1 point, 7, 1, 3 answer no 1 point, and 4 and 10 do not score. In order to reduce potential bias, the score is not included in the total score. Part B is to use a 128 Hz tuning fork and a 10 g monofilament to check vibration sense and light touch. This MNSI score is obtained by the diabetic patients filling in part A and professional physicians measuring part B, and the higher the score, the more severe the symptoms.

*(4) Quality of Life Scale for Patients with Type 2 Diabetes Mellitus (DMQLS)*. The Quality of Life Scale (DMQLS) suitable for Chinese patients with diabetes was adopted, which consists of 87 items in 5 dimensions: disease, physiology, society, psychology, and satisfaction. Among them, there are 20 items in the disease dimension, 17 items in the physiological dimension, 19 items in the social dimension, 16 items in the psychological dimension, and 15 items in the satisfaction dimension. The higher the score of each item, dimension, and total score, the more severe the patient's symptoms or function.

The article "Evaluation of Mindfulness Training Combined with Aerobic Exercise on Neurological Function and Quality of Life in Patients with Peripheral Neuropathy Type 2 Diabetes Mellitus" was published in 2022. Journal: Contrast Media Mol Imaging.

### 2.4. Statistical Approach

The EpiData3.1 software will be used to establish a database, and SPSS V.22.0 will be used for data processing and analysis. All statistical tests will be two-sided, with *α* = 0.05 considered as the test level. If the measurement data conform to the normal distribution, it will be described by a normal distribution; if it does not conform to the normal distribution, it will be described by the median and interquartile range. In the analysis of the results, if the data conformed to the normal distribution, the analysis of variance will be mainly used for statistical inference, and if the data did not conform to the normal distribution, the Wilcoxon Mann–Whitney rank sum test will be used for inference; count data will use Person's chi-square test. The graphing software used by the institute is GraphPad Prism 8.

## 3. Results

### 3.1. Comparison of SNCV and MNCV among the Three Groups

Before treatment, SNCV and MNCV were not significantly significant (*P* > 0.05), but after treatment, SNCV and MNCV were significantly higher, and the MMTC group changed more significantly (*P* < 0.05), as shown in Table 2 and Figure 1.

### 3.2. Comparison of MAAS and TCSS Scores among the Three Groups

Before treatment, MAAS and TCSS scores were not significant (*P* > 0.05); after treatment, MAAS scores were significantly higher, TCSS scores were significantly lower, and more significantly in MMTC, and they had a significant difference (*P* < 0.05), as shown in Table 3, and Figure 2.

### 3.3. Comparison of the Neurological Symptom Scores of the Three Groups

Before treatment, there was no statistical significance of the neurological sign score (*P* > 0.05). After treatment, the neurological symptom score and neurological sign score were significantly reduced, and the changes in the MMTC group were statistically significant (*P* < 0.05), as shown in Table 4 and Figure 3.

### 3.4. Comparison of QoL Scores among the Three Groups

There was no significant difference in the quality of life score before treatment (*P* > 0.05), and the quality of life score in the MMAE group was significantly increased (*P* < 0.05), as shown in Figure 4.

## 4. Discussion

Diabetic peripheral neuropathy is one of the most common types of diabetic neuropathy and one of the most common chronic complications of diabetes. Specifically, in the case of excluding other causes, diabetic patients have symptoms related to peripheral nerve dysfunction, and the clinical manifestations are symmetrical pain and paresthesia. T2DM is a chronic disease characterized by metabolic disorders and is often complicated by various complications [1]. T2DM adversely affects cardiovascular, renal, ocular, and neurological functions, and induces various complications. Diabetic peripheral neuropathy (DPN) is the most common complication of diabetes [2]. Diabetic patients have peripheral nerve dysfunction, of which distal symmetrical polyneuropathy (DSPN) is the most representative [3, 4]. According to the 2019 International Diabetes Federation (IDF) survey, there are 463 million people with diabetes (DM) worldwide, of which type 2 diabetes (T2DM) accounts for about 90%. The incidence of T2DM in China ranks the first in the world [5]. As the disease progresses, approximately 50% of DM patients are affected by DPN. In addition, approximately 10– 30 percent of patients with DPN experience neuropathic pain symptoms [6, 7]. The consequences of DPN can be devastating, with foot ulcers occurring in approximately 25% of patients with DPN [8], and it is the leading cause of lower extremity amputation in diabetes. In addition, many patients experience depression, sleep disturbance, and limited mobility due to the presence of DPN symptoms. It can even lead to a decline in the quality of life and disability of patients [9]. Therefore, timely intervention is essential to prevent the occurrence and development of DPN. At present, lifestyle intervention (mainly including exercise and diet) is recognized as an effective treatment method for DPN patients in addition to blood sugar control and drug therapy [10]. Drug therapy is currently used to relieve symptoms, but there are no drugs approved by the Food and Drug Administration (FDA) for the prevention or treatment of DPN in humans. The American Diabetes Association (ADA) guidelines state that moderate-intensity aerobic exercise can improve metabolism, microcirculation, and neurological function in patients with DPN, but there is a disagreement on how to choose an appropriate form of exercise for patients with DPN. Patient compliance is often poor if exercise therapy is used alone to intervene [11]. According to the fearavoidance model (FAM), physical discomfort and limitation of daily activities in patients with DPN can affect their social skills [12]. This may lead to adverse emotions such as anxiety and depression in patients, which can affect glycemic control and increase the incidence of complications [13]. Therefore, it is particularly urgent to explore physical and mental intervention methods suitable for DPN patients.

The article "Evaluation of Mindfulness Training Combined with Aerobic Exercise on Neurological Function and Quality of Life in Patients with Peripheral Neuropathy Type 2 Diabetes Mellitus" was published in 2022. Journal: Contrast Media Mol Imaging.

Aerobic exercise is also an important part of mind-body medicine. A lot of evidence shows that aerobic exercise is widely used in the prevention and treatment of diseases of different systems such as the respiratory system, circulatory system, and nervous system. Aerobic exercise movements are gentle. The waist is used as the axis when exercising [14]. The upper body performs a circular motion with the help of the spine. Lower the center of gravity of the lower body and stand with alternating legs. This puts muscles and related tissues throughout the body in a regular alternating state of contraction and relaxation. Therefore, the blood circulation and metabolism of the body are improved. It also has a positive effect on muscle strength, limb coordination, flexibility, and balance of exercised individuals. Aerobic exercise emphasizes concentration and mentally visualizes the movement. This allows the brain to focus on body sensations and also makes the proprioceptive system more sensitive. Mindfulness training is at the forefront of contemporary cognitive behavioral therapy. It can effectively relieve physical and mental illness while improving well-being. Mindfulness meditation focuses on developing a conscious, moment-to-moment, nonjudgmental awareness of experience. It helps to enhance attention to current experiences, including thoughts, sensations, breathing, and bodily sensations [14, 15]. DPN is the leading cause of foot ulcers and amputations in people with diabetes. Although diagnosis is easy, treatment is not very effective. Therefore, most patients experience pain during treatment. Mindfulness meditation can enable patients to more objectively assess discomfort and improve self-regulation, which can facilitate patient acceptance of the uncomfortable experience [16, 17]. If patients receive exercise therapy alone, patient compliance is often poor.

Previous studies have shown that adding mindfulness training to exercise effectively increases patients' willingness to exercise, increases the time and frequency of exercise, and promotes patients' perception of body sensations during exercise [18, 19]. At the same time, it can broaden the patient's vision and enhance their own understanding. It also helps the body become more flexible, relaxed, and balanced. Therefore, the negative experience of the patient is effectively alleviated. Mindfulness training focuses on improving the trainer's concentration while regulating breathing and relaxing the body [20]. This concept of mindfulness training is very much in line with the idea of aerobic exercise, and mindfulness meditation combined with aerobic exercise practice is more effective than aerobic exercise practice alone in improving clinical symptoms and neurological function in patients with DPN. Patients must be instructed to adjust their breathing while practicing Aerobic exercise [21, 22]. In addition, it is also important to instruct the patient to feel the pressure and relaxation of the alternate contraction and relaxation of the muscles of the legs, to experience the sensation of the feet touching the ground, and to encourage the patient to pay attention to his heart and learn to accept and relax. The patient obtains peace of mind and body, which is more conducive to improving the trainer's attention to the physical sensation of each movement, and the training effect is significantly improved. This study analyzed the changes in neurological function of patients before and after treatment. The results showed that there was no significant difference in various indicators before treatment (*P* > 0.05), but after treatment, patients' neurological function was significantly improved, and the quality of life was greatly improved. The findings of other scholars are highly consistent.

The article "Evaluation of Mindfulness Training Combined with Aerobic Exercise on Neurological Function and Quality of Life in Patients with Peripheral Neuropathy Type 2 Diabetes Mellitus" was published in 2022. Journal: Contrast Media Mol Imaging.

The research focuses on the effects of mindfulness training combined with Tai Chi on the neurological function and quality of life in patients with type 2 diabetic peripheral neuropathy. The topic is novel and can provide a good foundation for the patients' subsequent rehabilitation training. However, this study also has certain shortcomings because the included sample is small and the research period is short, which will affect the accuracy of the research results. Therefore, more eligible samples need to be included in the next study.

## 5. Conclusions

In summary, mindfulness training combined with aerobic exercise has an ideal therapeutic effect on patients with type 2 diabetic peripheral neuropathy and has a very important role in improving the neurological function and quality of life of the patients. It is a safe and effective treatment method. Therefore, mindfulness training combined with aerobic exercise therapy is worthy of promotion and application.

## Figures and Tables

**Figure 1:** Comparison of SNCV and MNCV in the three groups.

**Figure 2:** Comparison of MAAS and TCSS scores among the three groups.

**Figure 3:** Comparison of neurological symptom scores among the three groups.

**Figure 4:** Comparison of QoL scores among the three groups.

**Table 1:** The plan of type 2 diabetic peripheral neuropathy subjects based on “meta-awareness” mindfulness training combined with aerobic exercise.

Week	Project	Time	Training content
Week 1	Awareness and autopilot model		Introduce the rules of the course and pay attention to aerobic exercise
		1st time	Aerobic exercise, establishes a good relationship with patients, and discusses with patients the problems encountered in the self-management of type 2 diabetic peripheral neuropathy and related pain, coping strategies, and the concept and role of mindfulness
		2nd time	Aerobic exercise (integrate mindfulness into aerobic exercise and experience the feeling of the body during aerobic exercise) + somatosensory scan
		3rd time	Aerobic exercise (integrate mindfulness into aerobic exercise) + somatosensory scan, mindful breathing exercise (experience the in and out of gas), mindfulness meditation (awareness of inner activities) combined with the patient's pain and negative emotions to guide the subjects to make a reasonable reaction

Week 2	Live in ideas		Aerobic exercise + body scan, mindful breathing, and introducing mindfulness, joy, recognition thinking, and direct perception experience calendar into daily life
		4th time	Aerobic exercise (integrating mindfulness into aerobic exercise) + independent mindfulness awareness and experience and applying mindfulness to subjects' eating and activities
		5th time	Aerobic exercise (integrating mindfulness into aerobic exercise) + independent mindfulness awareness and experience, and applying mindfulness to subjects' lives
		6th time	Aerobic exercise (integrate mindfulness into aerobic exercise) + review previous exercises, summarize, and ask patients to share their insights from mindfulness practice

Week 3	Focus on the present moment	7th–9th time	Aerobic exercise (integrate mindfulness into aerobic exercise) + share happiness

Week 4	Learn to accept and let go	10th–12th time	Aerobic exercise (integrate mindfulness into aerobic exercise) + experience with difficulties

Week 5	Identify wrong thoughts	13th–15th time	Aerobic exercise (integrating mindfulness into aerobic exercise) + knowing yourself

Week 6	Ideas are not the same as facts	16th–18th time	Aerobic exercise (integrating mindfulness into aerobic exercise) + focus on breath, thoughts, body, and mood

Week 7	How to adjust yourself when you encounter difficulties	19th–21st time	Aerobic exercise (integrate mindfulness into aerobic exercise) + face up to physical discomfort and inner difficulties

Weeks 8 to 12	Maintenance training	22nd–36th time	Aerobic exercise (incorporating mindfulness into aerobic exercise)

The article "Evaluation of Mindfulness Training Combined with Aerobic Exercise on Neurological Function and Quality of Life in Patients with Peripheral Neuropathy Type 2 Diabetes Mellitus" was published in 2022. Journal: Contrast Media Mol Imaging.

**Table 2:** Comparison of SNCV and MNCV among the three groups.

Group	SNCV (m/s)				MNCV (m/s)			
	Nervi medianus		Nervus peroneus communis		Nervi medianus		Nervus peroneus communis	
	Pretreatment	Posttreatment	Pretreatment	Posttreatment	Pretreatment	Posttreatment	Pretreatment	Posttreatment
MM group	34.25 ± 1.83	37.52 ± 2.41	28.92 ± 1.23	34.22 ± 1.68	37.26 ± 1.42	40.36 ± 1.85	30.52 ± 2.36	35.42 ± 2.75
AE group	35.21 ± 1.92	39.52 ± 2.82	28.96 ± 1.22	35.47 ± 1.72	37.75 ± 1.54	40.26 ± 1.96	30.47 ± 2.54	38.72 ± 2.41
MMAE group	34.68 ± 1.82	43.51 ± 3.57	28.74 ± 1.25	39.41 ± 1.86	38.59 ± 1.55	43.57 ± 2.05	30.75 ± 2.65	43.68 ± 3.14
*F*	0.425	16.524	1.824	18.741	0.482	16.725	1.892	18.745
*P*	>0.05	<0.05	>0.05	<0.05	>0.05	<0.05	>0.05	<0.05

**Table 3:** Comparison of MAAS and TCSS scores among the three groups.

Group	MAAS (scores)		TCSS (scores)	
	Pretreatment	Posttreatment	Pretreatment	Posttreatment
MM group	46.52 ± 5.38	68.24 ± 6.52	11.25 ± 2.01	7.52 ± 1.68
AE group	46.51 ± 5.42	70.63 ± 6.89	11.24 ± 2.06	6.52 ± 1.42
MMAE group	46.58 ± 5.72	74.53 ± 6.82	11.19 ± 2.03	4.86 ± 1.17
*F*	1.865	17.425	0.429	18.472
*P*	>0.05	<0.05	>0.05	<0.05

The article "Evaluation of Mindfulness Training Combined with Aerobic Exercise on Neurological Function and Quality of Life in Patients with Peripheral Neuropathy Type 2 Diabetes Mellitus" was published in 2022. Journal: Contrast Media Mol Imaging.

**Table 4:** Comparison of the neurological symptom scores of the three groups.

Group	Neurological symptom score (score)		Neurological signs score (score)	
	Pretreatment	Posttreatment	Pretreatment	Posttreatment
MM group	6.02 ± 2.43	4.53 ± 0.85	1.92 ± 0.29	1.38 ± 0.14
AE group	5.92 ± 2.38	3.75 ± 0.57	1.89 ± 0.32	0.86 ± 0.15
MMAE group	5.24 ± 2.17	2.17 ± 0.34	1.91 ± 0.33	0.51 ± 0.17
*F*	0.527	20.635	1.411	19.754
*P*	>0.05	<0.05	>0.05	<0.05

## Data Availability

Data are available upon request from the corresponding author.
